# Intensive Health Care plus Vitamin D Administration Benefits the Growth and Development of Young Children and Reduces the Incidence of Nutritional Disorders

**DOI:** 10.1155/2022/8097035

**Published:** 2022-06-06

**Authors:** Yangyang Liu, Qingwen Zeng

**Affiliations:** ^1^Children Rehabilitation Department of Shiyan Maternal and Child Health Care Hospital, Shiyan, Hubei Province, China; ^2^Children Healthcare Center of Shiyan Maternal and Child Health Care Hospital, Shiyan, Hubei Province, China

## Abstract

This study was intended to assess the effect of intensive health care plus vitamin D administration on the growth, development, and nutritional status of young children. Totally, 131 young children who were admitted to Shiyan Maternal and Child Health Care Hospital from January 2020 to January 2021 were included and assigned via the random number table method at a ratio of 1 : 1 : 1 to receive either vitamin D administration (vitamin D group, *n* = 42), intensive health care (IHC) (IHC group, *n* = 44), or vitamin D administration plus intensive health care (combination group, *n* = 45). All children received a normal diet and routine care. After the intervention, all children showed robust improvement in their height, weight, neuropsychological development, and nutritional status, in which the combination therapy was associated with better outcomes in terms of physical development, neuropsychological development, and nutritional status, and a higher serum 25-hydroxyvitamin D3 (25-(OH)D3) level of the children versus monotherapy. Children receiving combined therapy had a significantly lower incidence of nutritional disorders than those receiving single therapy. Intensive health care plus vitamin D benefits the growth and development of young children and reduces the incidence of nutritional disorders in children.

## 1. Introduction

Childhood is a stage of rapid body growth, during which proper nutritional supply is of great significance. A previous study has demonstrated that a sufficient and reasonable nutritional supply is vital for children's physical growth and the development of cognitive, immune, and body functions [1]. Vitamin D is an essential nutrient element for children's growth and development. It regulates calcium and phosphorus metabolism and promotes tooth development and bone growth [2]. The 2016 edition of “Dietary Guidelines for Chinese Residents” [3] recommended that appropriate vitamin D administration within a few days after birth contributes to lowering the incidence of various diseases. Child health care is an important measure to protect children's physical and mental health and promote their growth [4]. Recent research has found that reasonable nutritional intervention yields a promising effect on children's health and cognitive development [5]. Accordingly, the concept of intensive health care is proposed, which, compared with conventional child health care, follows regular pediatric care and provides targeted health education and guidance on the growth and nutritional status of children. In addition, traditional Chinese medicine (TCM) plays an important role in strengthening health care. Research showed that TCM massage and acupoint massage can also promote children's growth and development [6]. A prior study has stated that intensive health care is associated with a lower incidence of nutritional disorders in children [7]. Therefore, this study analyzed the effects of intensive health care combined with vitamin D on the growth and nutritional status of young children, to constitute more effective child health care programs and promote the growth and nutritional status of children. The report is as follows.

## 2. Materials and Methods

### 2.1. Clinical Data

A total of 131 young children who were admitted to the children's health department of Shiyan Maternal and Child Health Care Hospital from January 2020 to January 2021 were included and randomly divided into the vitamin D group (*n* = 42), intensive children's health care group (ICH group) (*n* = 44), and combination group (*n* = 45). The study was approved by the hospital ethics committee, and the children (no. 2019-34/231) and their legal guardians signed an informed consent form.

### 2.2. Inclusion and Exclusion Criteria

#### 2.2.1. Inclusion Criteria

Children aged 0–6 years, with complete clinical data, who completed all interventions and follow-ups, with adequate physical examination results were included.

#### 2.2.2. Exclusion Criteria

Children with congenital or genetic diseases, with nutritional disorders diagnosed before enrollment, with premature birth, with hearing and intellectual impairments that prevented treatment cooperation were excluded.

### 2.3. Methods

All children in the group received a normal diet and routine child care. The vitamin D group received vitamin D administration, the IHC group received intensive health care, and the combination group received both vitamin D administration plus intensive health care. (1) Vitamin D administration: patients received 400 IU of oral vitamin D drops (Qingdao Shuangjing Pharmaceutical Co. Ltd., Approval No. H20113033) daily. (2) Intensive health care: targeted health education and guidance with regard to the growth, development, and nutritional status of the children were formulated and performed. (1) Disease prevention: the knowledge and prevention measures of nutritional diseases were introduced to the children's parents, and the children received regular disease screening and timely vaccination. (2) Early education: the instruction, training, and development of children's language, perception, and behavioral functions were strengthened. (3) Nutrition guidance: breastfeeding was encouraged, supplementary foods could be gradually added 6 months after birth, and foods rich in vitamins were given after complete weaning. Picky eating was timely corrected to achieve a balanced nutrition intake. (4) Parent health education: online or offline training was regularly held to improve the quality of parenting. (5) TCM health care: at the age of 18 months and 24 months, acupoint massage was performed on the Yingxiang and Zusanli points, and at the age of 30 months and 36 months, acupoint massage was performed on the Sishencong point.

### 2.4. Observational Indicators

#### 2.4.1. Baseline Characteristics

Children's age, gender, birth weight, birth height, birth season, feeding method, supplementary feeding time, and body mass index (BMI) were collected.

#### 2.4.2. Evaluation of Growth and Development

The children's height and weight were measured before the intervention, 3 months and 6 months after the intervention to calculate the BMI. The “0–6 Years Old Children's Neuropsychological Development Checklist” was used to assess the neuropsychological development of the children. The scale includes 5 aspects of adaptability, major movements, fine movements, language, and social interaction, with a total score of 100 points. The higher the score, the better the development in the corresponding aspect.

#### 2.4.3. Assessment of Nutritional Status

The venous blood of children was collected before the intervention, 3 months and 6 months after the intervention, and centrifuged at 3000 r/min for 5 minutes, to separate the serum for detection. The automatic biochemical analyzer (Siemens, Germany, model Atellica CH930) was used to determine the levels of hemoglobin (Hb) and albumin (ALB). The right upper arm circumference (in cm) was measured and repeated 3 times to obtain the average value.

#### 2.4.4. Serum 25-(OH)D3 Level

The venous blood of children was collected before the intervention, 3 months and 6 months after the intervention, and centrifuged to separate the serum for assay. An enzyme-linked immunosorbent assay was used to determine the level of (25-(OH)D3). The kits were purchased from Nanjing Senbega Biotechnology Co. Ltd. (Cat. No. SBJ-H1130). The experiments all employed kits with the same batch number.

#### 2.4.5. Occurrence of Nutritional Diseases

All children were followed up for six months, and the occurrence of children's vitamin D deficiency rickets, nutritional anemia, malnutrition, and diarrhea was recorded.

### 2.5. Statistical Methods

All the obtained data are analyzed using the SPSS20.0 software, and the GraphPad Prism 8.0 software was adopted to draw the figures. The measurement data conforming to the normal distribution are represented by (mean ± standard deviation), the independent sample *t*-test was used for intergroup comparison, the paired sample *t*-test was used for intragroup comparison, the single factor analysis of variance was used for the three-group comparison, and the Snk-*q* test was used for pairwise comparison. The counting data are expressed as frequency or composition ratio. If the total number of cases was less than 40 or the minimum theoretical frequency was less than 1, the chi-square exact probability method was used. If the total number of cases was ≥40 and the minimum theoretical frequency was 1∼5, the chi-square correction method was used. If the total number of cases was greater than or equal to 40 and the minimum theoretical frequency was greater than 5, the chi-square noncorrection method was used. *P* < 0.05 indicates that the difference is statistically significant.

## 3. Results

### 3.1. Comparison of Baseline Data

There were 42 cases in the vitamin D group, including 21 males and 21 females, aged 0–6 years old, with an average age of 3.35 ± 0.42 years. There were 44 cases in the vitamin D group, including 24 males and 20 females, aged 0.5–6 years, with an average age of 3.38 ± 0.46 years. There were 45 cases in the vitamin D group, including 23 males and 22 females, aged 0.5–6 years, with an average age of 3.32 ± 0.44 years. There was no statistically significant difference in age, birth weight, birth height, birth BMI, gender, birth season, feeding method, and supplementary feeding time of the three groups of children (*P* > 0.05) (Table 1).

### 3.2. Comparison of the Physical Development

Children in the three groups showed similar height and weight before the intervention (*P* > 0.05). After the intervention, the height and weight of the children in the three groups increased significantly compared with those before the intervention (*P* < 0.05). The differences in the height and weight of the children between the vitamin D group and the IHC group were not statistically different (*P* > 0.05), while the combination group had better results than the other two groups (*P* < 0.05), as shown in Table 2.

### 3.3. Comparison of Neuropsychological Development

The three groups presented no great disparity in the neuropsychological development before the intervention (*P* > 0.05). After the intervention, the neuropsychological development of the three groups of children showed a marked improvement (*P* < 0.05), with the best results observed in the combination group than the other two groups (*P* < 0.05), and the neuropsychological development of the vitamin D group and the IHC group was similar (*P* > 0.05) (Table 3).

### 3.4. Comparison of Serum 25-(OH)D3 Levels

Before the intervention, the three groups showed similar serum 25-(OH)D3 levels (*P* > 0.05). After the intervention, the combination group showed better outcomes in terms of physical development, neuropsychological development, and nutritional status, and a higher serum 25-(OH)D3 level of the children than the other two groups (*P* < 0.05), as shown in Figure 1.

### 3.5. Comparison of the Nutritional Status

Before the intervention, the three groups had no significant difference in nutritional status (*P* > 0.05). After the intervention, the nutritional status of the three groups of children was all significantly improved (*P* < 0.05), the combination group achieved the greatest enrichment in the nutritional status of the children than the other two groups (*P* < 0.05), and the nutritional status of the vitamin D group and the IHC group was similar (*P* > 0.05). (Table 4).

### 3.6. Comparison of the Occurrence of Nutritional Diseases

The incidence of nutritional diseases in children in the combination group was significantly lower than in the other two groups (*P* < 0.05) (Table 5).

## 4. Discussion

Currently, the concept of childcare extends from simple physical health care to comprehensive care for neuropsychological development [8, 9]. Traditional childcare mainly includes height and weight measurement and cardiopulmonary examination, but its effect is unsatisfactory [10, 11]. Intensive health care provides additional nutritional interventions, disease prevention and screening, and early health education guidance. Previous research has suggested that individualized nutrition guidance contributes to promoting children's growth and development and improving their nutritional status [12], and that health education on nutrition and hygiene knowledge for children's family members contributes to optimizing the children's dietary structure and enhancing their nutritional status [13]. Vitamin D deficiency is directly linked to serious complications in children, leading to rickets, fetal growth restriction, and eczema [14]. The high prevalence of vitamin D deficiency [15] has drawn the attention of professionals to the development of related preventive measures [16].

This study compared the effects of vitamin D administration, intensive health care, and vitamin D administration plus intensive health care on the growth and development and nutritional status of young children. The results of the present study showed that after the intervention, the height and weight of the children in the three groups increased significantly compared with those before the intervention. The height and weight of the children in the vitamin D group and the IHC group were not statistically different, while the combination group had better results than the other two groups, indicating that compared with a single intervention, a targeted combined therapy regimen is more conducive to the physical development of children. Previous research has found that vitamin D plays a key role in maintaining the normal physiological functions of children's neuropsychiatric system [17], and that child health interventions and nursing strategies benefit the neuropsychological development of infants and young children [18]. The results of the present study demonstrated that the neuropsychological development of children after the intervention was significantly improved compared with that before the intervention, with better outcomes observed in children receiving combined therapy, which was in line with the results of previous studies. Serum 25-(OH)D3 is the main active form of vitamin D in the body. The results of this study found that the serum 25-(OH)D3 levels of children in the vitamin D group and the combination group after the intervention were higher than before the intervention, but there was no significant change in the IHC group, which was consistent with previous research results, suggesting that intensive health care combined with vitamin D administration enhance the absorption of vitamin D by the body, thereby promoting the regulation of calcium and phosphorus metabolism. Despite the availability of natural sources of vitamin D to increase 25-(OH)D3 levels, these sources are generally considered ineffective in maintaining 25-(OH)D3 levels in the 30–50 ng/mL (75–125 nmol/L) range year-round. Adverse effects associated with vitamin D use, such as hypercalcemia and hypercalciuria, are rare and are usually caused by prolonged use of extremely high doses of vitamin D, which indicated a high safety profile of vitamin D administration [19]. Moreover, this study used Hb, ALB, and upper arm circumference to assess the nutritional status of children and found that after the intervention, the nutritional status of the children in the three groups was markedly enhanced compared with that before the intervention, with better results observed in the combination group, indicating that targeted nutritional intervention and appropriate vitamin D administration contributes to optimizing the nutritional supply of children and effectively reducing the incidence of nutritional disorders. Previous study has confirmed that a concentration of 25(OH)D ≥ 30 ng/mL is associated with higher hemoglobin levels, which is essential for children's growth and development [20].

## 5. Conclusion

Intensive health care plus vitamin D benefits the growth and development of young children and reduces the incidence of nutritional diseases in children.

## Figures and Tables

**Figure 1:** Comparison of serum 25-(OH)D3 levels in three groups of children.

**Table 1:** Comparison of baseline data of three groups of children.

Items	Vitamin D group (*n* = 42)	IHC group (*n* = 44)	Combination group (*n* = 45)	*F*/*χ*^2^	*P* value
Age (year)	3.35 ± 0.42	3.38 ± 0.46	3.32 ± 0.44	0.206	0.814

Birth weight (kg)	3.34 ± 0.28	3.41 ± 0.24	3.28 ± 0.27	2.708	0.071

Birth length (m)	0.51 ± 0.12	0.53 ± 0.15	0.47 ± 0.13	2.311	0.103

Birth BMI (kg/m^2^)	13.23 ± 1.24	13.27 ± 1.26	13.32 ± 1.21	0.058	0.944

Gender				0.195	0.907
Male	21	24	23		
Female	21	20	22		

Birth season				5.048	0.538
Spring	8	10	15		
Summer	9	13	12		
Autumn	11	12	9		
Winter	14	9	9		

Feeding method				2.136	0.983
Breast milk	28	25	31		
Artificial feeding	6	10	8		
Combined feeding	8	9	6		

Supplementary feeding time				0.509	0.775
<6 months	29	31	34		
≥6 months	13	13	11		

**Table 2:** Comparison of physical development of children in three groups ($\bar{x}\pm s$).

Groups	*n*	Time points	Height (m)	Weight (kg)
Vitamin D group	42	Before intervention	0.71 ± 0.17	11.34 ± 1.23
		3 months after intervention	0.93 ± 0.18^③^	14.98 ± 1.19^③^
		6 months after intervention	1.16 ± 0.21^③④^	17.36 ± 1.25^③④^
		*F*	62.377	265.588
		*P* value	<0.01	<0.01

IHC group	44	Before intervention	0.68 ± 0.19	11.28 ± 1.25
		3 months after intervention	0.89 ± 0.17^③^	14.92 ± 1.21^③^
		6 months after intervention	1.13 ± 0.18^③④^	17.31 ± 1.23^③④^
		*F*	68.120	263.767
		*P* value	<0.01	<0.01

Combination group	45	Before intervention	0.73 ± 0.15	11.24 ± 1.26
		3 months after intervention	0.98 ± 0.14^①②③^	15.79 ± 1.23^①②③^
		6 months after intervention	1.24 ± 0.17^①②③④^	18.83 ± 1.25^①②③④^
		*F*	119.325	406.355
		*P* value	<0.01	<0.01

Compared with the vitamin D group at the same time point, ^①^*P* < 0.05; compared with the IHC group at the same time point, ^②^*P* < 0.05; compared with the same group before intervention, ^③^*P* < 0.05; compared with the same group after 3 months of intervention, ^④^*P* < 0.05.

**Table 3:** Comparison of the neuropsychological development of the three groups of children (points, $\bar{x}\pm s$).

Groups	*n*	Time points	Adaptability	Majormovements	Finemovements	Language	Social interaction
Vitamin D group	42	Before intervention	69.22 ± 4.34	70.12 ± 3.98	66.28 ± 3.42	71.22 ± 2.17	62.39 ± 3.48
		3 months after intervention	80.93 ± 4.37^③^	82.29 ± 4.12^③^	76.15 ± 3.36^③^	80.39 ± 1.96^③^	67.56 ± 3.45^③^
		6 months after intervention	92.76 ± 4.42^③④^	91.16 ± 4.23^③④^	87.87 ± 3.37^③④^	89.87 ± 2.14^③④^	73.92 ± 3.41^③④^
		*F*	303.735	285.501	444.613	864.693	122.378
		*P* value	<0.01	<0.01	<0.01	<0.01	<0.01

IHC group	44	Before intervention	68.78 ± 4.42	69.34 ± 3.94	67.11 ± 3.47	71.45 ± 2.14	63.28 ± 3.51
		3 months after intervention	81.46 ± 4.39^③^	84.81 ± 4.15^③^	77.43 ± 3.34^③^	81.28 ± 2.03^③^	68.13 ± 3.47^③^
		6 months after intervention	93.88 ± 4.45^③④^	92.76 ± 4.24^③④^	88.11 ± 3.23^③④^	90.32 ± 2.16^③④^	74.26 ± 3.43^③④^
		*F*	354.730	369.106	432.789	879.637	110.627
		*P* value	<0.01	<0.01	<0.01	<0.01	<0.01

Combination	45	Before intervention	68.95 ± 4.38	69.58 ± 3.95	66.57 ± 3.38	71.36 ± 2.15	62.89 ± 3.42
		3 months after intervention	86.52 ± 4.34^①②③^	87.98 ± 4.21^①②③^	83.56 ± 3.41^①②③^	85.79 ± 2.13^①②③^	74.82 ± 3.41^①②③^
		6 months after intervention	96.74 ± 4.47^①②③④^	96.49 ± 4.25^①②③④^	94.61 ± 3.35^①②③④^	95.65 ± 2.17^①②③④^	81.26 ± 3.38^①②③④^
		*F*	459.862	497.000	785.780	1452.770	337.513
		*P* value	<0.01	<0.01	<0.01	<0.01	<0.01

Compared with the vitamin D group at the same timepoint, ^①^*P* < 0.05; compared with the IHC group at the same timepoint, ^②^*P* < 0.05; compared with the same group before the intervention, ^③^*P* < 0.05; compared with the same group after 3 months of intervention, ^④^*P* < 0.05.

**Table 4:** Comparison of nutritional status of children in three groups ($\bar{x}\pm s$).

Groups	*n*	Time point	Hb (g/L)	ALB (mg/L)	Upper arm circumference (cm)
Vitamin D group	42	Before intervention	108.32 ± 3.89	31.78 ± 1.73	10.42 ± 1.28
		3 months after intervention	116.76 ± 3.76^③^	35.46 ± 1.79^③^	13.58 ± 1.24^③^
		6 months after intervention	121.24 ± 3.73^③④^	39.23 ± 1.84^③④^	15.91 ± 1.32^③④^
		*F*	125.579	25.923	194.500
		*P* value	<0.01	<0.01	<0.01

IHC group	44	Before intervention	109.14 ± 3.92	31.45 ± 1.85	10.25 ± 1.26
		3 months after intervention	115.36 ± 3.73^③^	36.31 ± 1.76^③^	14.13 ± 1.21^③^
		6 months after intervention	122.45 ± 3.69^③④^	38.84 ± 1.82^③④^	16.12 ± 1.35^③④^
		*F*	136.482	189.364	241.351
		*P* value	<0.01	<0.01	<0.01

Combination group	45	Before intervention	108.74 ± 3.95	31.44 ± 1.76	10.37 ± 1.24
		3 months after intervention	121.49 ± 3.67^①②③^	38.94 ± 1.73^①②③^	15.98 ± 1.23^①②③^
		6 months after intervention	129.86 ± 3.74^①②③④^	44.79 ± 1.78^①②③④^	19.85 ± 1.27^①②③④^
		*F*	354.633	652.954	657.701
		*P* value	<0.01	<0.01	<0.01

Compared with the vitamin D group at the same time point, ^①^*P* < 0.05; compared with the IHC group at the same timepoint, ^②^*P* < 0.05; compared with the same group before the intervention, ^③^*P* < 0.05; compared with the same group after 3 months of intervention, ^④^*P* < 0.05.

**Table 5:** Comparison of the occurrence of nutritional diseases among the three groups of children (*n* (%)).

Groups	*n*	Vitamin D deficiency rickets	Nutritional anemia	Malnutrition	Diarrhea	Total
Vitamin D group	42	4	3	2	2	11
IHC group	44	4	2	3	3	12
Combination group	45	1	0	1	0	2
*χ* ^2^	9.530					
*P* value	0.009					

Compared with the vitamin D group at the same time point, ^①^*P* < 0.05; compared with the intensive health care group at the same timepoint, ^②^*P* < 0.05; compared with the same group before the intervention, ^③^*P* < 0.05; compared with the same group after 3 months of intervention, ^④^*P* < 0.05.

## Data Availability

The data used to support the findings of this study are available from the corresponding author upon request.
